# A Widow-Maker and a Doppelganger: An Anomalous Case of the Coronaries

**DOI:** 10.7759/cureus.9603

**Published:** 2020-08-07

**Authors:** Jahanzeb Malik, Tayyaba Zahid, Omaid Majedi, Uzma Ishaq, Muhammad Ishfaq Faizi

**Affiliations:** 1 Cardiology, Rawalpindi Institute of Cardiology, Rawalpindi, PAK; 2 Hematology and Medical Oncology, Foundation University/ Fauji Foundation Hospital, Rawalpindi, PAK

**Keywords:** "anomalous coronary artery", st-elevation myocardial infarction (stemi), primary percutaneous coronary intervention, left main stem thrombus, dual left anterior descending artery, lms clot, coronary artery bypass grafting(cabg), anomalous left circumflex artery

## Abstract

The anomalous origin of the left circumflex (LCX) artery from the right coronary sinus is a relatively rare condition. A ‘double’ left anterior descending (LAD) artery is probably the rarest of coronary artery anomalies. We present a case of acute myocardial infarction with a clot and a critical distal stenosis in the left main stem (LMS) supplying a dual LAD and an aberrant origin of the LCX.

## Introduction

Coronary artery anomalies are rare and diverse congenital disorders with varying presentations and mechanisms. Most of the aberrations do not affect the quality of life. However, the presence of certain anomalous presentations is an important pathological entity that should be evaluated as they can cause myocardial infarction (MI) or sudden cardiac death (SCD) [1]. The overall incidence of an anomalous coronary artery is around 1.2% [2]. Aberrant left circumflex (LCX) arising from the right coronary sinus is frequently seen but ‘double’ left anterior descending artery (LAD) is only present in 1% of the population [3, 4].

We present a case of a middle-aged gentleman showing up as an acute MI. On invasive angiography, he was found to have a couple of coronary abnormalities and a clot in the left main stem (LMS).

## Case presentation

A 52-year-old man presented at our institute with an hour of severe, central, and crushing chest pain with nausea and diaphoresis. He gave no history of any comorbid conditions except a strong family history of ischemic heart disease. His older brother had a myocardial infarction a couple of years ago. On examination, his heart rate was 100 beats/min, the rhythm was sinus. Blood pressure was 160/100 mmHg. The chest was clear to auscultate and no added sounds were present on precordial examination.

His electrocardiogram (ECG) was done which showed ST-elevation in the chest leads V2 to V6 (Figure 1). He was diagnosed as an anterior MI.

**Figure 1:** Electrocardiogram of the patient showing regular sinus rhythm, normal axis and ST-segment elevation in the precordial leads (V2 - V6)

The first set of Troponin I was 0.3 ng/ml (negative up to 0.4 ng/ml). Baseline hematology and biochemistry were normal. Echocardiogram showed anterior and apical hypokinesia of the left ventricle (LV). He was loaded with 300 mg and 600 mg of Aspirin and clopidogrel, respectively. The subcutaneous injection of heparin (5000 U) was administered while he was moved to a cardiac catheterization laboratory. His coronary angiogram was done showing the unusual findings (Figures 2-4).

**Figure 2:** (A) Antero-posterior view of the left system showing a thrombus in the left main stem (red arrow) and a critical disease distally (black arrow) continuing as a left anterior descending artery. (B) Right anterior oblique view showing the thrombus (red arrow) and a critical distal disease (black arrow). The left main stem continues as a left anterior descending artery which divides into the dual left anterior descending arteries in the middle.

**Figure 3:** 30-degree left anterior oblique view showing non-dominant right coronary artery which appears to be disease-free.

**Figure 4:** (A, B) Right anterior oblique and antero-posterior views showing an aberrant left circumflex artery arising from right coronary sinus instead of the left coronary system. The vessel appears to be disease-free.

The LMS was not bifurcating and had a distal critical disease before continuing as LAD. There was a thrombus visible in the mid-course. The continuation was a dual LAD system bifurcating into two distinct arteries at the middle, supplying the middle anterior, and the lateral wall of the LV. Upon cannulating the right coronary artery (RCA), a shadow of an aberrant LCX artery can be seen. RCA was non-dominant and normal. For the LCX, a multipurpose catheter was engaged and views taken.

After completion of the angiogram, a lead surgeon was called to review the coronary anatomy. It was mutually decided to keep the patient on tirofiban infusion. The case was discussed regarding further intervention in a heart team meeting. After explaining the risks and benefits, he was counseled regarding his future outcome. The patient opted for a coronary artery bypass grafting (CABG).

After a five-day stay at a surgical ICU, he was discharged on Aspirin and clopidogrel 75 mg daily. Guideline-directed medical therapy was started for acute coronary syndrome (ACS). After a month’s follow-up, the patient was doing well.

## Discussion

Coronary artery anomalies are defined as an abnormal coronary pattern not observed or very rare among the general population. About 1/3rd of the coronary anomalies involve aortic root pathology or asymmetry of the aortic sinuses [5]. Although anomalous coronary anatomy is rare, it is the second major cause of sudden cardiac death among the athletes [6].

There are three elements of coronary vasculature which are crucial to their development: (1) the sinusoids, (2) the vascular endothelial network, (3) the coronary buds on the aortic sinus. The coronary arteries develop within the atrioventricular and interventricular grooves with their proximal parts arising from the aortic valve sinuses [7]. There is a direct relationship between the distribution, the coronary size, and the extent of their dependant myocardium. Abnormalities in the development of the coronary buds are implicated in coronary artery anomalies [7].

The anomalous origin of the LCX from the right coronary sinus was first described in 1933. It can arise from RCA or a separate ostium. It is seen in 0.67% of the patients and in the absence of atherosclerotic disease, it is considered benign [8]. This was the case in our patient. The dual LAD has been reported to occur in various case reports and case series. There are four types of dual LADs defined in the literature [9]. Our patient did not fall in any of the four categories as both the divisions supplied different areas of the myocardium. The only clue towards the double nature of the LAD was that both branches are giving off septal perforators. The presence of anomalous coronary anatomy does not confer an elevated risk for atherosclerotic coronary artery disease but the patients can sometimes present with an acute coronary syndrome.

Left main coronary erosion or rupture of an atherosclerotic plaque with thrombus formation is the leading cause of death with the mortality of two- to three-fold greater than patients with one- or two-vessel disease [10]. Our patient had an atherosclerotic plaque rupture leading to thrombus formation and propagation into the left-main. This is an indication of a coronary intervention either with stenting or CABG. However, there are mixed opinions about either of the approaches regarding unprotected left main disease. NOBEL and EXCEL are the most notable of all the trials which have demonstrated contemporary percutaneous coronary intervention (PCI) to be non-inferior to CABG [11, 12]. In contrast, the SYNTAX trial showed that CABG conferred less major adverse cardiovascular events when compared with PCI [13]. Our patient underwent CABG after a heart team discussion and he was the decision-maker for his procedure.

## Conclusions

Coronary artery anomalies should be regarded as the rare and diverse group of congenital abnormalities with variable outcomes. Most of these aberrancies are benign while others confer an increased risk of MI or SCD. Atherosclerotic unprotected left main disease is best managed by CABG, particularly in young patients with a favorable long-term survival and safety.
